# Artificial Fuzzy-PID Gain Scheduling Algorithm Design for Motion Control in Differential Drive Mobile Robotic Platforms

**DOI:** 10.1155/2021/5542888

**Published:** 2021-10-18

**Authors:** Najah Yousfi Allagui, Farhan A. Salem, Awad M. Aljuaid

**Affiliations:** Industrial Engineering Department, College of Engineering, Taif University, P.O. Box 11099, Taif 21944, Saudi Arabia

## Abstract

Mobile robots are promising devices which are dedicated to human comfort in all areas. However, the control algorithm of the wheels of mobile robot is entirely challenging due to the nonlinearity. Recently, the classical PID (proportional-integral-derivative) controllers are frequently used in robotics for their high accuracy and the smooth determination of their parameters. A robust approach called fuzzy control which is based on the conversion of linguistic inference sets in a suitable control value is a widely used method in industrial system control in our days. A new challenging method to solve the problem of intelligent navigation of nonholonomic mobile robot is suggested. In this work, the presented methodology is based on three hybrid fuzzy logic PID controllers which are adapted to guarantee target achievement and trajectory tracking. A fuzzy-PID control algorithm is designed with 2 inputs and 3 outputs. By the information given by the system response, error and error derivate can be used to extract and adopt the PID controller parameters: proportional, integral, and derivative gains. Besides, a tuning value A is introduced to improve the resulted response in terms of speeding up and reducing error, overshoot, and oscillation, as well as reducing ISE and IAE values. A modelization of a differential drive mobile robot is presented. The developed algorithm is tested and implemented to this mobile robot model via Simulink/MATLAB.

## 1. Introduction

Mobile robots have been a crucial element of our modernized life. Robots can be described as intelligent machines that can facilitate many activities in different areas such as industry, medical, military, and family services. The ability of robot to perform tasks with potential risks in an unknown environment is considered as a strong characteristic due to the incapability of humans to reach some hazardous regions and targets. In robotic research, one of the most important matters is motion control, which is how to make the robot to track or to navigate from a start point to a desired target without collision with obstacles. By reason of existence of motion planning in practically all mobile robotics applications, researchers are concerned by different control approaches of mobile robots.

The design process of mobile robotic platforms is not a simple task; as a whole, the process consists of various stages and aspects, in particular, the platform design, the electric motor sizing, control algorithm design, modeling, and verification process. Beside all this, and due to the fact that the mobile robot is a time variant system, there are various factors that affect the design process, including the platform's operational parameters; the surrounding environment and the road conditions are always varying.

In the field of mobile robotic platforms design, one of the most important design tasks is the motion problem. This problem is categorized into three categories: navigation, path following, and trajectory tracking. The control algorithm plays an important role in the working ability of mobile robotic platform; therefore, the overall mobile robot system with its subsystems and components must be designed to be robust and adaptive system, as well as operates with improved dynamic and with a good steady state system performances [1].

Research on PID controllers is a very big challenging area that attracts many scientists. Large number of methods and approaches are discussed for years. An optimal robust PID controller is developed using future search algorithm which is dedicated to systems with uncertain parameters [2]. This controller demonstrates a good stability and robustness [2].

Another approach-based bacterial foraging optimization algorithm is well used to extract the optimized parameters of PI controller in order to be applied to an electrical grids system. This approach gives a best performance compared to the classical genetic algorithm approach [3]. For the design of a shipper controller to energy management instead of the expensive classical solutions, a novel approach-based fuzzy sliding mode was developed in order to maintain the frequency output under its limit and ensure system stability for systems with uncertainties [4].

The problem of nonlinearity was discussed and treated in a lot of papers. Different control methods were used to solve this problem like improved neural networks control system applied to a robotic manipulator [5]. The problem of controlling nonlinear systems is also resolved by other approaches such as fuzzy logic controller and fuzzy-PID controllers.

The majority of industrial control approaches are based on conventional control method like PID by cause of its reliability and simplicity. Unfortunately, the PID controllers present some drawbacks like the reduction of PID performances towards nonlinear systems. Also, applying PID algorithm stability and tracking can be achieved, but not accuracy. Other controlling approaches like the famous FLC (fuzzy logic controller) are presented as an alternative of classical PID controller. These controllers-based artificial fuzzy logic algorithm gained significant popularity in the last years. Fuzzy algorithm can be designed to propose solutions for solving motion problem including performing path planning, local navigation, global navigation, steering control, and rate control of a mobile robot [6, 7].

The FLC controller uses human reasoning to produce a suitable output with respect to eventual limitations. These controllers are widely used to produce control outputs for complex and/or nonlinear systems, thanks to its capability to handle with heuristic and imprecise information. The flexibility of FLC to establish nonlinear control algorithms is a well-known argument to use these algorithms, especially in motion control and tracking of mobile robots [1, 6–11].

Fuzzy-PID control design, the controller that mixes the PID with fuzzy logic systems, is called the hybrid fuzzy-PID controller. Fuzzy logic PID control design is the process of adjusting the parameters of the PID controller adopting the fuzzy logic. The online tuning of parameters of PID controller-based fuzzy logic systems makes it more compliant [12, 13].

Large number of researchers are interested by the advantageous hybrid fuzzy-PID controller in different areas like controlling DC motor speed, hydroxy generators, and synchronous motors [12–16]. An improved dynamic response with short response time, smooth overshoot, and a low SSE error are perceived and confirmed by them [12–16]. The flexibility of fuzzy logic controller as well as the simplicity of PID algorithms are exploited to guarantee a good path tracking of our mobile robot.

The main contribution in this presented study is the adoption of hybrid fuzzy-PID-based dynamic model to control a nonholonomic WMR (wheeled mobile robot). The effort in this paper is demonstrated in the modelization as well as the extraction of the dynamic model of our robot. A novel parameter A is added in the flowchart of hybrid fuzzy-PID gain scheduling algorithm. This great parameter allows overcoming some drawbacks like oscillations in robot motion curvature. Also, a software prototype model for mobile robot platform is advanced. The importance of this prototype is to testify the developed approach in different design stages; in particular, this can help designers to identify mobile robot system level problems at fresh design stage. The developed platform ensures design modifications process and helps in solving the motion control problem in terms of assessing designed control algorithm for achieving desired output motion aspects. The designed hybrid fuzzy logic controller is developed and applied to a mobile robot dynamic model and, finally, validated via the performed software platform.

Fuzzy-PID gain scheduling algorithm for path tracking is to be designed and tested. The work is written as follows: in Section 2, system methodology and working principle are presented. In Section 3, modeling of mobile robotic system is included. In Section 4, the hybrid fuzzy-PID gain scheduling algorithm design is presented. In Section 5, testing, results, and discussion are presented; finally, in Section 6, conclusions and future work are given.

## 2. System Methodology and Working Principle

The structure of the direct action fuzzy algorithm with two inputs and one output is shown in Figure 1(a). There are different types of fuzzy algorithm structures; in this work, the applied hybrid fuzzy-PID control algorithm type is the artificial hybrid fuzzy-PID gain scheduling algorithm; the structure of this algorithm is shown in Figure 1(b). In this algorithm structure type, depending on system error value, the controlled system response state, and the effect of each of PID gains *K*_*P*_, KI, and *K*_*D*_ on system response, the knowledge base and fuzzy inference engine are developed and used to assign the values of the conventional PID gains online. The final control signal, to drive the controlled system, is still generated by the conventional PID algorithm [8, 9].  Figure 1(c) shows flowchart representation of the fuzzy algorithm working principle and PID gain calculations. Meanwhile, representing using block diagrams of the overall mobile robotic platform system motion control with components layout is shown in Figure 1(d).

## 3. Modeling of Mobile Robotic System

In the literature, modeling of mobile robot system can be found in different sources, including [10, 11, 17–21].

In MATLAB/Simulink environment, a software prototype model for mobile robotic platform is developed. The prototype is developed to help the designers in different design stages, in particular, identifying mobile robot system level problems at early design stage, design modifications process, and ensuring that all design specifications and requirements are met, in addition to help in solving the motion control problem in terms of assessing designed control algorithm for achieving desired output motion aspects. The software prototype model shown in Figure 2(d) was built considering the factors that affect the design process including the mobile robot operational parameters, the working environment, and the road/path conditions. The prototype is developed by integrating the models of the next subsystem: electric machines, kinematics, dynamics, odometry, sensors, control algorithms, as well as modeling the data readings and inputting components, and the performance indices modeling. These models shown in Figure 2 are built to result in maximum output data in graphical and numerical forms. Beside numerically displayed values, the built software prototype returns the next graphical data: platform's angular and linear speeds, linear speeds of left and right wheels, the robot orientation direction, and the curvature covered distance, in addition to this, left and right wheels positions and curvature. Moreover, the software prototype is developed to return the data needed to assess both the sizing of the electric motor and the design control algorithm and, finally, the electric motor's response in terms of the consumed current and performance indices to achieve desired linear speed under given load torques.

In the next paragraph, the equation and mathematical models used to represent subsystems and build Simulink submodels are summarized: the resultant force of all the acting forces on a running mobile robotic platform is the sum of all acting forces and is given by equation (1). This resultant force is converted to torque by the robot's wheels, axels, and speed as given by equation (2). The linear velocities of the two left *υ*_*L*_ and right *υ*_*R*_ wheels can be calculated in terms of mobile robotic platform angular speed as by equation (3). In this equation, *R* is the distance between two points, the ICC point and the midpoint P, between the two wheels. *R* can be found by equation (4). The curvature, which is the inverse of the radius *R,* gives equation (5). The angular velocity of the platform can be represented by equation (6). The platform instant linear velocity *v*_mob_ is calculated by equation (7). The two components of linear velocities in *x*-axis and *y*-axis direction are given by equation (8). The mobile platform angular position can be found as by equation (9). The overall mobile robot platform system based on the electric DC motor system, which can be represented in transfer function form with gear ratio, *n*, is given by equation (10). The power driver (amplifier) circuit with gain *K*_*a*_ can be represented by transfer function given by equation (11):

(1) $$\begin{array}{c} F_{\text{Total}}=F_{\text{aerod}}+F_{\text{rolling}}+F_{\text{climb}}+F_{\text{angl}\_\text{acc}}+F_{\text{lin}\_\text{acc}}+F_{\text{wind}}, \end{array}$$

(2) $$\begin{array}{c} T_{\text{Load}}=r*F_{\text{Total}}, \end{array}$$

(3) $$\begin{array}{c} \upsilon_{L}=\omega_{\text{mob}}\left(R+\frac{L}{2}\right), \end{array}$$

(4) $$\begin{array}{c} R=\frac{\upsilon_{R}+\upsilon_{L}}{\upsilon_{R}-\upsilon_{L}}*\frac{L}{2}, \end{array}$$

(5) $$\begin{array}{c} \lambda =\frac{1}{R}=\frac{\omega }{\upsilon_{\text{mob}}}=\frac{2}{L}*\frac{\left(\upsilon_{R}-\upsilon_{L}\right)}{\left(\upsilon_{R}+\upsilon_{L}\right)}, \end{array}$$

(6) $$\begin{array}{c} \omega =\frac{\upsilon_{R}-\upsilon_{L}}{L}=\frac{\left(\omega_{R}-\omega_{L}\right)r}{L}, \end{array}$$

(7) $$\begin{array}{c} \upsilon_{\text{mob}}=\frac{\upsilon_{R}+\upsilon_{L}}{2}=\frac{\left(\omega_{R}+\omega_{L}\right)r}{2}, \end{array}$$

(8) $$\begin{array}{c} \upsilon_{x}=\upsilon_{mob}\sin\left(\theta \right)=\frac{\left(\omega_{R}+\omega_{L}\right)r}{2}\sin\left(\theta \right)=\frac{\upsilon_{R}+\upsilon_{L}}{2}\sin\left(\theta \right), \end{array}$$

(9) $$\begin{array}{c} x\left(t\right)=\int \left(\frac{\upsilon_{R}+\upsilon_{L}}{2}\right)\sin\left(\theta \left(t\right)\right)dt+x_{0}, \end{array}$$

(10) $$\begin{array}{c} G_{\text{speed}}\left(s\right)=\frac{\omega_{\text{robot}}\left(s\right)}{V_{\text{in}}\left(s\right)}= \end{array}$$

(11) $$\begin{array}{c} G\left(s\right)=\frac{K_{a}}{\text{0.}01\text{s}+1}, \end{array}$$

## 4. Hybrid Fuzzy-PID Gain Scheduling Algorithm Design

The proposed hybrid fuzzy gain scheduling algorithm is developed based on the following works [7, 22–24].

The rule base look-up tables for calculating and relating the PID gain values are listed as Tables 1–3. To develop the knowledge from the rule base and built inference engine, the applied rule inference method is the Mamdani method, and the used defuzzification approach was the centroid method [7, 24]. To express the knowledge levels and represent linguistic variable, triangular membership functions are selected.

The linguistic variables used are NB, NS, Z0, PS, PB, VB, B, M, and S. The ranges of universes of discourse are selected as follows: for *e*, [−2, 2], Δ*e*, [−3, 3], and *K*_*P*_, [−1, 1], for *K*_*D*_, [−0.1, 0.1], and for *K*_*I*_, [−0.05, 0.05]. In case the resulted overall system response requires further improvement, in terms of speeding up response and reducing each of the resulted overshoot, oscillation, and error, as shown in Figure 3(a), a single tuning parameter A is used for scaling the system error value. Tuning the value of this parameter will improve the resulted response in terms of speeding up and reducing error, overshoot, and oscillation, as well as reducing ISE and IAE values.

The Simulink models representing the developed fuzzy-PID algorithm submodel and the PID algorithm sub-block are shown in Figures 3(b) and 3(c). The designed artificial fuzzy algorithm in MATLAB/Simulink in terms of membership function with linguistic variables and their universe of discourse ranges are shown in Figure 4(d).

## 5. Testing, Results, and Discussion

Figure 2 shows an integrated mobile platform software simulation prototype model which is employed to test and assess both the designed hybrid fuzzy algorithm and system responses, and the robotic system is tested for achieving various robot tracking motion profiles. The utilized motor electric and dimensional parameters to be used in the simulation and testing process are listed in Table 4.

The presented tests are discussed as follows:

- Test (1): testing the control algorithm for motion tracking in terms of achieving straight line motion with desired linear speed of 0.5 m/s. Beside numerically displayed values listed in Tables 5–7, the software prototype returns the overall robotic system and subsystems responses in graphical data curve forms, as depicted in Figures 4(a)–4(d). Analyzing the resulted data in numbers and graphical forms show that the robotic system achieved desired linear speed of 0.5 m/s, with acceptable performance measure. To further improve the resulted response and reduce oscillation and overshoots, the tuning parameter A is tuned to have the values of 0.02765.
- Test (2): Test (2) is depicted to test the mobile robotic platform using the designed control algorithm; for turning to the right, the left motor is subjected to a signal with 5% decrease compared to the right one. So, the right motor speed is decreased to 0.475 m/sm, while the left motor speed is remained to be 0.5 m/s; this result is numerically displayed in Tables 5–7, and response curves are depicted in Figures 4(a)–4(d). Analyzing the resulted data shows that the robotic system turned to the left direction with linear speed of 0.4875 m/s and angular speed of 0.0625 rad/s. The robotic system tracked the desired motion path, as shown in Figures 5(a)–5(d), with turning radius of −7.8 m, curvature of −0.1282, and orientation direction of −1.63 degrees.
- Test (3): Test (3) is dedicated to test the ability of the system to follow a straight line motion, with a desired linear speed from 0 to 3 m/s, and this speed is maintained for a specific time and finally reduced to attain zero; these results are numerically displayed in Tables 5–7 and response curves are depicted in Figure 6. Analyzing the resulted data shows that the robotic system followed the desired motion profile, but with some oscillation. As a remedy to this oscillation, a soft tuning of parameter A (decreasing) can be applied which will remove this effect.

It is concluded after the analysis of these tests that the nonholonomic mobile robot followed its desired motion profile with acceptable performance measures. However, some oscillations are depicted which are removed by the soft tuning parameter A.

The proposed control methodology presents some advantages such as simplicity in design, assured stability, and optimal and precise control specifications that are proved by the convergence of the tracking error to a minor value. Simulation and experimental ensured by developed platform verified the sufficient and consistent results in path tracking.

## 6. Conclusions

The classical PID controllers presented many limitations like accuracy and the initial condition problems are overcome by the hybrid fuzzy-PID controller. A strong design of a hybrid fuzzy-PID controller is suggested in this work to perform robot navigation and tracking. A trajectory tracking is achieved using the hybrid fuzzy-PID controller which presents efficient results. Both circular and straight line paths are tested to demonstrate the utility of the developed motion control approach. A new parameter A is introduced in the flowchart of hybrid fuzzy-PID gain scheduling algorithm. This strong parameter allows overcoming some drawbacks like oscillations in robot motion curvature. A developed differential drive mobile robotic platform is presented with a detailed modelization. The mobile robot prototype is developed by integrating the models of the next subsystem: electric machines, kinematics, dynamics, odometry, sensors, control algorithms, as well as modeling data readings and inputting components, and the performance indices modeling. This platform is used to test and evaluate the designed algorithm based on Simulink/MATLAB. An implementation of the obtained control design methods via the developed mobile robot platform is discussed for three different types of tests: Test (1): testing the control algorithm for motion tracking in terms of achieving straight line motion with desired linear speed of 0.5 m/s; Test (2): testing the mobile robotic platform, using designed control algorithm, for turning to the right by subjecting the left motor to signal with 5% less than the right one; and Test (3): testing the system to follow a straight line motion but with motion profile to reach desired linear speed from zero to 3 m/s. Sufficient and consistent results in path tracking are obtained which confirm the utility of combined fuzzy and PID control approach. Based on these findings, as future works, some algorithms of optimization like particle swarm optimization or genetic algorithms will be exploited to adapt the fuzzy-PID parameters, and developing the motion control approaches in dynamic environment will be our objective in future works. Besides, we will be interested by the nonholonomic mobile robot with two different motors to discuss with details the problem of stability of robot motion recently in progress.

## Figures and Tables

**Figure 1:** (a) Fuzzy algorithm structure. (b) The system architecture of fuzzy-PID gain scheduling algorithm. (c) The flowchart representation of hybrid fuzzy-PID gain scheduling algorithm. (d) Representing the overall mobile robotic platform system motion control with components layout.

**Figure 2:** (a) Simulink submodel of electric DC motor and torques consisting of acting forces in running robotic system. (b) Model for generating different input signal types. (c) Simulink model for reading and evaluating the performance indices. (d) An overall one integrated mobile robotic system software simulation model.

**Figure 3:** (a) The hybrid fuzzy-PID algorithm with one tuning input factor A for tuning the error value. (b) The Simulink model representing the developed fuzzy-PID algorithm submodel. (c) The PID algorithm sub-block. (d) The fuzzy algorithm with two inputs and four outputs in MATLAB/Simulink. (e) Error-related membership function, linguistic variables, and universe of discourse range. (f) Rate of error-related membership function, linguistic variables, and universe of discourse range. (g) Membership function with linguistic variables and their universe of discourse ranges for assigning *K*_*P*_ values. (h) Membership function with linguistic variables and their universe of discourse ranges for assigning *K*_*i*_ values. (k) Membership function with linguistic variables and their universe of discourse ranges for assigning *K*_*D*_ values.

**Figure 4:** (a) Test (1): the resulted robot straight line motion with linear speed of 0.5 m/s. (b) Test (1): robotic system response curves representing robot's linear speed, angular speed, and curvature. (c) Test (1): robotic system response curves representing robot's desired and actual linear speeds, right and left wheel position, and turning radius. (d) Test (1): robotic system response curves representing robot's orientation direction, and performance indices values in terms of ISE and IAE of both wheels.

**Figure 5:** (a) Test (2): the resulted robot circular motion with left motor 5% desired speed less than the right one. (b) Test (2): robotic system response curves representing robot's linear speed, angular speed, and curvature. (c) Test (2): robotic system response curves representing robot's desired and actual linear speeds, right and left wheels position, and turning radius. (d) Test (1): robotic system response curves representing robot's orientation direction and performance indices values in terms of ISE and IAE of both wheels.

**Figure 6:** Test (3): robotic system response curves representing robot's linear speed, angular speed, and curvature for tracking motion profile.

**Table 1:** Fuzzy rules table for assigning the *K*_*p*_.

Δ*e*	Error				
	NB	NS	ZO	PS	PB
NB	VB	VB	S	S	M
NS	VB	B	S	S	B
ZO	B	M	S	S	VB
PS	M	S	S	M	VB
PB	S	S	S	B	VB

**Table 2:** Fuzzy rules table for assigning the *K*_*D*_.

Δ*e*	Error				
	NB	NS	ZO	PS	PB
NB	S	S	VB	B	S
NS	S	S	B	B	S
ZO	S	M	B	M	S
PS	M	B	B	S	S
PB	M	B	VB	S	S

**Table 3:** Fuzzy rules table for assigning the *K*_*I*_.

Δ*e*	Error				
	NB	NS	ZO	PS	PB
NB	S	M	M	M	S
NS	B	B	B	B	B
ZO	B	B	BV	VB	VB
PS	B	B	B	B	B
PB	S	S	M	M	S

**Table 4:** Electric DC motor subsystem parameters.

Parameter	Unit
Torque constant, Kt	1,1882 Nm/A
Armature resistance, Ra	0.1557 Ohms (Ω)
Armature inductance, La	0.82 MH
Geared-motor inertia, Jm	0.271 kg.m^2^
Motor viscous damping, *b*_m_	0.271 N.m.s
Motor back EMF constant, kb	1.185 rad/s/v
Gear ratio	*n* = 3
The aerodynamic drag coefficient, Cd	0.80
The air density (*kg/m*^3^) at STP, *ρ*	1.25
Wheel radius, r	0.075 m
Platform height, h	0.920 m
Platform width, b	0.580 m
Wheels center distance	0.4 m
Total platform mass	100 kg
Total equiv. inertia, Jequiv	0.2752 kg.m^2^
Total equiv. damping	0.3922 N.m.s
The coefficient of lift, CL	0.13
Inclination angle to be	45 degrees

**Table 5:** Testing results, data for response analysis.

	Desired speed	Actual speed	Error	Overshoot	Settling time	5T	Current, SS	Control signal, SS	ISE	IAE
Test (1)	L: 0.5	L: 0.5	L: 0	L: 0	L: 11	L: 13	L: 5.764	L: 0.5836	L: 58.6	L: 19.59
	R: 0.5	R: 0.5	R: 0	R: 0	R: 11	R: 13	R: 5.764	R: 0.5836	R: 58.6	R: 19.59

Test (2)	L: 0.475	L: 0.475	L: 0	L: 0	L: 11.5	L: 13.4	L: 5.482	L: 0.5546	L: 49.59	L: 17.18
	R: 0.5	R: 0.5	R: 0	R: 0	R: 11.5	R: 13.4	R: 5.764	R: 0.5836	R: 58.6	R: 19.59

**Table 6:** Testing results, overall mobile robotic platform.

	Tuning parameter A	Platform linear speed	Platform angular speed	Left wheel linear speed	Right wheel linear speed	Left wheel angular speed	Right wheel angular speed
Test (1)	0.02765	0.5	0	0.5	0.5	6.667	6.667
Test (2)	0.3	0,4877	−0.062525	0.4752	0.5	6.333	6.667

**Table 7:** Testing results, overall mobile robotic platform (2).

	Platform curvature	Platform turning radius	Left wheel curvature	Right wheel curvature	Robot orientation direction
Test (1)	0	Inf	Inf	Inf	0
Test (2)	−0.1282	−7.799	−7.999	−7.5999	−0.326

## Data Availability

Data are available on request to the corresponding author.
